The article "Histopathological and clinical evaluation of Kombucha tea and Nitrofurazone on cutaneous full-thickness wounds healing in rats: an experimental study" was retracted in 2016. Reasons: misconduct by an author; plagiarized text; compromised peer review; false authorship.

# Histopathological and clinical evaluation of Kombucha tea and Nitrofurazone on cutaneous full-thickness wounds healing in rats: an experimental study

**DOI:** 10.1186/1746-1596-8-120

**Published:** 2013-07-17

**Authors:** Fardin Barati, Javad Javanbakht, Farajollah Adib-Hashemi, Ehsan Hosseini, Reyhaneh Safaeie, Mojtaba Rajabian, Mostafa Razmjoo, Reza Sedaghat, Mehdi Aghamohammad Hassan

**Affiliations:** 1 Department of Clinical Science, Faculty of Veterinary Medicine, Tehran University, Tehran, Iran; 2 Department of Pathology, Faculty of Veterinary Medicine, Tehran University, Tehran, Iran; 3 Faculty of Para Veterinary Medicine, Ilam University, Ilam, Iran; 4 Gradaute, Faculty of Veterinary Medicine, Tehran University, Tehran, Iran; 5 Food Hygiene Department, University of Shahekord, Shahekord, Iran; 6 Faculty of Veterinary Medicine, Razi University, Kermanshah, Iran; 7 Department of Pathology, Faculty of Medicine Science, Shahed University, Tehran, Iran

**Keywords:** Wound healing, Kombucha fungus, Nitrofurazone, Histopathological, Clinical

## Abstract

**Background:**

Kombucha, a fermented tea (KT) is claimed to possess many beneficial properties. The aim of this study was to evaluate clinical and histopathological alterations of Kombucha tea and Nitrofurazone on cutaneous full-thickness wounds healing in rat.

**Methods:**

In present study 24 Wister -albino rats weighing 150–200 g were selected and divided to two treatment groups as Nitrofurazone ointment (0.2%) and Kombucha tea. Subsequently, the anesthesia was exerted by Ketamin hydrochloride 10% (40 mg/kg) and Xylasine (2 mg/kg) through intra muscular (IM) route. Furthermore, upon preparation of dorsal region of the animal for surgery, a piece of full-thickness skin removed (2 × 2 cm). In order to comparing wounds healing clinically and histologically, once every four days from the commencement, the wounds were photographed and the healed surface was measured by Scion image software.

**Result:**

The clinical findings indicated that the Kombucha fungus resulted in precipitating healing than Nitrofurazone; however, it was not significant (p > 0.05). In order to pathological comparing of wound healing process, several wound biopsies were taken on 4, 8, 12, 16 and 20^th^ days. Additionally, the histopathological results demonstrated that there was inflammation in Nitrofurazone group through twelveth day, somehow the epithelium was formed and abundant vessels were visible. Although on 16^th^ day and the previous days the healing condition of Kombucha fungus was considered as minimal rate, revealing it is similar to Nitrofurazone group on 20^th^ day.

**Conclusions:**

To wrap up. These observations suggest that the Kombucha fungus healing quality was rapid from 12^th^ day to the end of the research, whereas no significant difference was observed.

The article "Histopathological and clinical evaluation of Kombucha tea and Nitrofurazone on cutaneous full-thickness wounds healing in rats: an experimental study" was retracted in 2016. Reasons: misconduct by an author; plagiarized text; compromised peer review; false authorship.

**Virtual slide:**

The virtual slide(s) for this article can be found here: http://www.diagnosticpathology.diagnomx.eu/vs/1107407136102196

## Background

The wound healing process is a normal physiological response to injury and generally leads to restoration of normal structure and function in damaged tissues. In certain disorders, the wound healing process leads to an altered restitution of tissue structure and function that is associated with the development of remodeling and fibrosis [1,2].

Kombucha is a traditional beverage consumed in various parts of the world and especially in Asia. Its earliest known use originated with Dr. Kombu in 220 BC for curing the digestive troubles of Japan’s emperor. Many health promoting effects of Kombucha have been claimed [3], but adverse effects attributed to this beverage have been reported as well [4]. Kombucha is typically prepared by fermenting black tea, sweetened with sugar, with what is popularly known as a ‘tea fungus,’ at room temperature for 10–12 days [5,6]. This so called ‘tea fungus’ is actually a symbiosis of yeasts and acetic acid bacteria, the cellulosic pellicle formed by the latter commonly described as the ‘fungus’ [7-9].

Currently, Kombucha is alternately praised as “the ultimate health drink” [9,10] or damned as “unsafe medicinal tea” [10-12]. Testimonials claim causal benefits for everything from AIDS improvement, balding relief, cancer cures, and diabetic and arthritic symptom relief to prolonged longevity, weight loss, and cognition enhancements [13,14]. In conjunction with Kombucha’s growing popularity, life-threatening human health problems are beginning to be reported. Hepatotoxicity, [15] necrotizing pancreatitis, 16 and several human deaths have been linked to drinking Kombucha beverage [11,16,17].

In traditional medicine Kombucha was used for many disease treatments, including wound healing. Because of high abilities of Kombucha in curing, antibiotic, detoxification and skin luminosity it was supposed to determine the effect on injured skin in vitro condition. The composition and properties of tea are well documented, but scarce scientific information is available concerning the composition and the effects of Kombucha on health. Benefits have been reported by testimony of users in different conditions and with variable consummation. Nitrofurazone, an antibacterial drug was found to be photolabile; its photolability has been described in a number of recent papers [17,18].

Nitrofurazone is a synthetic nitrofuran with abroad antibacterial spectrum; it acts by inhibiting bacterialenzymes involved in carbohydrate metabolism [19]. Nitrofurazone is a topical anti-infective agent with a broadantibacterial spectrum; bactericidal against most bacteria commonly causing surface infections, including *S aureus, Streptococcus*[20].

The article "Histopathological and clinical evaluation of Kombucha tea and Nitrofurazone on cutaneous full-thickness wounds healing in rats: an experimental study" was retracted in 2016. Reasons: misconduct by an author; plagiarized text; compromised peer review; false authorship.

Wound healing is a dynamic process that involves the integrated action of a number of cell types (the interactions of many cells types, including inflammatory cells, fibroblasts, keratinocytes and endothelial cells, as well as the involvement of growth factors and enzymes), the extra cellular matrix, and soluble mediators termed cytokines. The normal adult healing process proceeds through a number of overlapping events: clot formation, inflammation, re-epithelialization, angiogenesis, granulation tissue formation, wound contraction, scar formation and tissue remodeling. Growth factors released in the traumatized area promote cell migration into the wound area (chemotaxis), stimulate the growth of epithelial cells, and fibroblasts (mitogenesis) initiate the formation of new blood vessels (angiogenesis) and stimulate matrix formation and remodeling of the affected region. The formation of new blood vessels from pre-existing capillaries that are then able to penetrate the wound site is an essential component of the wound healing process [21-23].

Until now, no knowledge has been available pertaining to the histological study of Kombucha tea treatment on wound healing in injured skin. The aim of the present study was to use histopathological and clinical methods to evaluate the effect of Kombucha tea and Nitrofurazone on cutaneous full-thickness wounds healing in rats.

## Methods

### Animals

All experimental protocols were approved by the local animal care committee in accordance with Faculty of Tehran Veterinary Medicine office regulations. In current study, 24 Wister -albino rats of both sexes, weighing 200–250 g, were utilized. The animals were kept in individual propylene cages under standard laboratory conditions by the dimensions of 30 × 50 × 25 cm^3^ two by two. Rats were maintained on a 12 hour light/dark cycle at 22 ± 1°C and 50 ± 10% humidity. The animals were kept in standard room conditions and fed with standard rat diet and water ad libitum.

### Preparation of Kombucha tea

Brooke Bond Red Label Tea (Hindustan Lever Limited, Mumbai, India) was used for the preparation of kombucha tea. Tea was added to boiling water (1.2%) and allowed to infuse for about 5 min after which the infusions were filtered through a sterile sieve. Sucrose (10%) was dissolved in hot tea, and the preparation was left to cool. The cooled tea (200 mL) was poured into 500 mL glass jars that had been previously sterilized at 121°C for 20 min and inoculated with 3% (w/v) freshly grown tea fungus that had been cultured in the same medium for 14 days and 10% (v/v) previously fermented liquid tea broth aseptically. The jar was covered with a clean cloth and fastened tightly. The fermentation was carried out in the dark at 24 3°C for 14 days [24,25].

The article "Histopathological and clinical evaluation of Kombucha tea and Nitrofurazone on cutaneous full-thickness wounds healing in rats: an experimental study" was retracted in 2016. Reasons: misconduct by an author; plagiarized text; compromised peer review; false authorship.

### Fermentation

Kombucha culture was kept under aseptic conditions. Fermentation was carried out by incubating the Kombucha culture at 28 ± 1°C for 8–10 days. Subsequently, the medium (brew) was centrifuged at 3000 rpm for 30 minutes aseptically and stored in polypropylene vials at -20°C for further use [26].

### Fractionation of Kombucha

Kombucha was subsequently fractionated using ethyl acetate (1:2, V/V). The solvent extracts and the remaining aqueous phase were concentrated using a vacuum rotary evaporator (R-200 model of Buchi Co, Germany). The obtained sticky mass was dissolved in distilled water appropriately and filtered through 0.22 μ Millipore membrane filter (Millipore Co, St-Quentin-en-Yvelines, France), later allowed to degas it. The concentrated extracts were freezed at -50°C to -60°C before subjecting to lyophilize and stored the lyophilized extract of kombucha at -20°C according to modified method of Jayabalan [24]. The lyophilization process was carried out at Orchid Pharmaceuticals, Chennai, India. The desired daily dose of lyophilized aqueous extract of kombucha was prepared with milli-Q-water as stock and reconstituted to different volumes with milli-Q-water as per designed doses just before subjecting to treatment.

### Surgical technique

In present study, a region as 4 × 4 cm was shaved after anesthesia and prepared for surgery following scrub. In addition, a piece of full-thickness (2 × 2 cm) skin was removed from dorsal surface of the animal using a sterile scalpel and a simple forceps, hence an open wound was created, the digital photography was implemented and finally the wound was bandaged by paraffin gauze dressing, wibril and adhesive plaster. Wounds were covered with sterile gauzes, which were fixed with adhesive tape (width, 4 cm) extending to the dorsal area. As described previously [27], Kombucha and Nitrofurazone ointment (0.1 mL) were applied to the wound surfaces. Next, all wounds were covered with sterile gauzes and fixed. The second treatment was performed 6 hours later and repeated 3 times per four day for 20 days [27].

### Experimental protocol

The rats were divided into two groups after 24 hours and randomly allotted into one of two experimental groups each group contains twelve animals, somehow each group was taken one of cures as a (Nitrofurazone 0.2%) and b (Kombucha fungus) and then were bandaged.

The article "Histopathological and clinical evaluation of Kombucha tea and Nitrofurazone on cutaneous full-thickness wounds healing in rats: an experimental study" was retracted in 2016. Reasons: misconduct by an author; plagiarized text; compromised peer review; false authorship.

### Photography

The photography of wounds was performed in order to clinical comparing of healing process of two treatment groups. The trend was started from the beginning and repeated every four days. For clinical assessment, the captured photos were analyzed by Scion image software which aimed to measure healing process and epithelialization, and were compared between two treatment groups as well. The measurement method was as transfer of scanned wound pictures into cited software, and measuring scale system, firstly, was chosen through known internal points in each figure and was calibrated for two vertical and horizontal directions. Consequently, by operating the software, the epithelial tissue edges were ascertained and located in suitable condition to account and recording it by the software.

### Sample collection and microscopic examination

In order to examining histopathological comparing of treatment effects on 4th, 8th, 12th and 20th days, the animals were killed under ether anesthesia. The hairs around the wound were shortened with scissors and removed with depilatory cream. The skin outside the wound was wiped with 70% ethanol and povidone-iodine. The sutures in closed wounds were removed. With a no 15 scalpel, approximately 3 cm^2^ rectangular tissue samples including epidermis, dermis, and subcutaneous tissue with 0.5 cm margin from wound edges and ends were taken. The mentioned method was performed following intra muscular injection of Ketamin hydrochloride 10% (high dose), and the samples were taken from dorsal region and healed tissue along with slightly of normal parts. In addition, the sample was fixed in a unolit by a disinfected needle, by povidine iodine, then tissue fragments were fixed in 10% neutral buffered formalin solution (for 72 hours), upon stability embedded in paraffin, sectioned at 5 μm thickness and stained with hematoxylin and eosin (H&E).

### Evaluation of inflammatory cell infiltration angiogenesis, fibroplasias and complete healing

Angiogenesis, fibroplasias, complete healing and inflammatory cell infiltration were evaluated in H&E-stained sections and scored semi quantitatively as follows: no or minimal angiogenesis, fibroplasias, complete and inflammatory cell infiltration (-), mild angiogenesis, fibroplasias and complete, inflammatory cell infiltration (+), inflammatory cells form extent and severity /moderate to severe angiogenesis, fibroplasias and complete (++), confluent inflammatory cell aggregates/moderate edema (+++) [26].

### Statistical analysis

The data were analyzed using the SPSS 7.5 Windows Students version software. For all the measurements, one-way ANOVA followed by Student’s–Newman–Keul’s (SNK) test was used to assess the statistical significance of difference between Nitrofurazone and Kombucha tea (lyophilized extract) treated. A statistically significant difference was considered at the level of *P* < 0.05.

The article "Histopathological and clinical evaluation of Kombucha tea and Nitrofurazone on cutaneous full-thickness wounds healing in rats: an experimental study" was retracted in 2016. Reasons: misconduct by an author; plagiarized text; compromised peer review; false authorship.

## Results

### Clinical findings

Upon analytical evaluation, the comparison of three variables such as wound contraction, epithelialization and complete healing of the wounds on 4^th^, 8^th^, 12^th^, 16^th^ and 20^th^ days in two treatment groups by Spss software using t-test was demonstrated that in Kombucha group the healing was faster which was significant (p < 0.05) in all cases, however. It should be notified that there was remarkable healing in benefit to Kombucha fungus during the performance at all three variables. Furthermore, the full healing (100%) was pertained to Kombucha treatment group though no considerable difference was recorded in Nitrofurazone group at all variables (Additional file 1 Chart 1 and 2).

### Histopathological findings

#### ***Extent and severity of the inflammation***

a. The inflammatory cells were not seen (^_^)

b. Observation of inflammatory cells at two microscopic fields (+)

c. Observation of inflammatory cells at 3–5 microscopic fields (++)

d. Observation of inflammatory cells at more than 5 microscopic fields (+++) (Tables 1 and 2)

**Table 1:** Histolopathological survey in the treatment group with Nitrofurazone

**Day 20**	**Day 16**	**Day 12**	**Day 8**	**Day 4**	**Circumstances wound healing progresses**
_	+	++	++	+++	Severity and extent of inflammation
+++	++	+	+	+	Fibroplasia
_	+	++	+++	+++	Angiogenesis
					
+++	+	+	+	_	Complete wound healing

**Table 2:** Histolopathological survey in the treatment group with Kombucha tea

**Day 20**	**Day 16**	**Day 12**	**Day 8**	**Day 4**	**Circumstances wound healing progresses**
_	_	++	++	+++	Severity and extent of inflammation
+++	++	++	+	+	Fibroplasia
_	+	+	++	++	Angiogenesis
+++	++	+	+	_	Complete wound healing

#### ***Angiogenesis***

a. The blood vessels were not seen (^_^)

b. Existing of 0–2 blood vessels (+)

c. Existing of 3–4 blood vessels (++)

d. Existing of more than 4 blood vessels (+++) (Tables 1 and 2)

#### ***Fibroplasia***

a. Recording of few thin collagen fibers along with numerous fibroblasts (^_^)

b. Recording of thin collagen fibers along with very numerous fibroblasts (+)

c. Recording of thick collagen fibers along with numerous fibroblasts (++)

d. Recording of abundant thick collagen fibers along with few fibroblasts (+++) (Tables 1 and 2)

### Complete wound healing

Emergence of thick collagen particles in harmony with slight fibroblasts and loss of blood vessels or inflammatory cells indicated the complete wound healing. According to pathological findings revealed that in two treatment groups by Nitrofurazone, the inflammation was observable through 12^th^ day as well as loss of epithelialization, but a large number of blood vessels were created (Figure 1 A, B, C and D). However, in Kombucha treatment groups the epithelialization was obvious on 12^th^ day and the trend was completely formed on 16^th^ day (Figure 2A, B, C and D). Overall, the healing condition at Kombucha treatment group was similar to Nitrofurazone on 20^th^ day; however, the results indicated which the Kombucha fungus healing enjoyed conspicuous clinically and histopathologically effects on 12^th^ day by the end of the research.

The article "Histopathological and clinical evaluation of Kombucha tea and Nitrofurazone on cutaneous full-thickness wounds healing in rats: an experimental study" was retracted in 2016. Reasons: misconduct by an author; plagiarized text; compromised peer review; false authorship.

**Figure 1:** **Histopatholigically, Nitrofurazone treatments groups are in different days. **A Four day inflammatory responses associated with intradermal immune infiltrates with promoting angiogenesis, B: Eighth day Excessive inflammation and angiogenesis during wound healing, C: Twelfth and sixteenth days; Loss of epithelial integrity associated with abundant angiogenesis and inflammation cells and epithelial tissues are formed by cells that cover the organ surface but not completed unlike Kumbucha, D: Twentieth day healing is crazy acceptable, closing up of the wounds with out inflammation and dermal appendages destroyed.

**Figure 2:** **Histopatholigically, Kumbucha treatment group in different days. A **Fourth day, Loss off epithelial associated with angiogenesis and inflammation, **B**: Eighth and twelfth day , loss of epithelial associated with abundant vessels and excessive inflammation and newly formed blood vessels and scarce amount of inflammatory elements, **C**: Sixteenth day, relatively good after healing after sixteenth day and dermal appendages destroyed, **D**: Twentieth day, Healing is crazy acceptable.

According to statistical analysis demonstrated that the inflammation severity on 8^th^, 4^th^ and 12^th^ days was severe in two treatment groups and showed no significant difference, whereas on 16^th^ day saw an remarkable difference (p < 0.05) at inflammation security rate which decreased in Kombucha group (Tables 1 and 2). However, it was the same with no any difference on 20^th^ day. The angiogenesis rate on 4^th^, 12^th^, 8^th^ and 16^th^ days was more in Nitrofurazone group than Kombucha group with no considerable difference and the angiogenesis was also the same in two groups on 20^th^ day (Figure 1A, B, C and D).The fibroplasias rate was the same on 8 and 9^th^ days although indicated no significant difference on 12^th^ at Kombucha group and it was the same on 16^th^ and 20^th^ days as well.

The article "Histopathological and clinical evaluation of Kombucha tea and Nitrofurazone on cutaneous full-thickness wounds healing in rats: an experimental study" was retracted in 2016. Reasons: misconduct by an author; plagiarized text; compromised peer review; false authorship.

The complete wound healing was the same and had no significant difference at two treatment groups (Additional file 1 Chart 1-4)). Accordingly, the complete wound healing at two treatment group was the same with no any significant difference, thus due to remarkable reduction of inflammation on 16^th^ day at Kombucha group, and no conspicuous rise regarding fibroplasia on 12^th^ day, revealed that the healing quality at Kombucha group was considered to be more beneficial (Figure 2A, B, C and D). On the other hand, it can be microscopically considered that the cause of more efficient healing of Kombucha group, that indicated no significant differences with Nitrofurazone group, was the severe reduction of the inflammation along with more fibroplasia on cited days which emerged positive effects on final contraction and epithelialization of the wound [28].

## Discussion

The wound healing is a complicated phenomenon, but regular, which some organized processes contribute in it. The human have being tested diverse chemical and herbal materials on wound healing [29,30] (Figure 3).

**Figure 3:** **Scheme of different stages of cutaneous wound repair in rats: A, B and C: The first 12- 24 hours after injury is defined by the platelet plug and blood clot formation.** Inflammatory cells invade the blood clot triggering acute inflammatory response. Furthermore, blood elements and vasoactive amines extravasate from locally damaged blood vessels within the dermis. Vascular permeability is temporarily increased to allow neutrophils, platelets and plasma proteins to infiltrate the wound. Coagulation then occurs as platelets aggregate with fibrin. **D, E and F**: After 48–72 h, macrophages replace polymorphonuclear neutrophils as the principal inflammatory cell. Together, polymorphonuclear neutrophils and macrophages remove debris from the wound, release growth factors, and begin to reorganise the extracellular matrix. The proliferation phase begins at about 72 h as fibroblasts, recruited to the wound by growth factors released by inflammatory cells, begin to synthesise collagen. The new tissue is called granulation tissue. Keratinocytes proliferate at the wound edge and migrate down the injured dermis and above the provisional matrix. 1–2 week after injury the wound is completely filled with granulation tissue. Fibroblasts have transformed into myofibroblasts, leading to wound contraction and collagen deposition. The wound is completely covered with a neoepidermis. Modified from Steven R. Beanes et el., 2003.

In present study, the results demonstrated faster healing by Kombucha than Nitrofurazone, but no significant difference was visible. According to histological finding revealed that at Nitrofurazone group inflammation, numerous blood vessels with no any epitheliogenesis were observable. Overall, the healing condition at Kombucha group was similar to Nitrofurazone on 20th day, whereas on 16th day and former days the healing considered as minimal.

The article "Histopathological and clinical evaluation of Kombucha tea and Nitrofurazone on cutaneous full-thickness wounds healing in rats: an experimental study" was retracted in 2016. Reasons: misconduct by an author; plagiarized text; compromised peer review; false authorship.

In addition, microscopical and histopathological factors ascertained that the healing quality of Kombucha fungus was more beneficial on 12th day by the end of the research; however, indicated no significant difference. Maghsoudi and Mohammadi in 2009 assessed the Kombucha influence on removing of postoperation intrapretoneal adhesion, and claimed that the cause was the oxidized treated cellulose and hyaluronic acid or its solution [31].

In a study by king in 2006 cited that high indication of hyaluronic acid during wound healing was rapid wound recovery and scar reduction [32]. Longaker et al., in 2008 indicated that HA reduces 5–10 days after injury [33]. Therefore, the increase of such fundamental material during wound healing, utilization of the colony of enriched HA termed Kombucha, could be advantageous. Topham in 2002 demonstrated that the embryonic ulcers recover without any scar and become full of HA as embryonic extracellular matrix [34]. In addition, Locono et al., 2005 cultured the forelimb of embryos in vitro and triggered an ulcer on it, hence finally indicated that the external HA decreased wound [35]. Lee et al., 1995 found that the HA induces fibroblast proliferation which produced efficient locomotor forces for wound contraction [36]. Furthermore, Weigel in 1986 ascertained that the minor particle of HA stimulates phagocytosis of macrophages [37]. Prohibiting of macrophage function postpones the healing process. Moreover, the source of HA, existing in Kombucha, reservoir has being accessed through microorganism fermentation. Of other effective compound in wound healing is vitamin C which has been observed in Kombucha as well.

Krichner et al., 2003 demonstrated that such vitamin precipitated the wound recovery in postoperative patients [38]. Jagetia et al., 2004 indicated that the wound improvement delay due to γ rays attributed to Ascorbic acid decrease and believes that the vitamin C increased the collagen content and vessels intensity, somehow such rise is indispensable for tissue damages and for wounds in remodeling phase [39]. Prashant et al., 2008 through microscopic cellulose assessment of Kombucha, originating from fermentation, found that such material carry beneficial effect on promoting chronic ulcer healing as ulcers with venous origin, bed sore and diabetics ulcers with difficult remedies [40]. Brown and Chem, 1886 reported that Acetobacter Xylinum generates stiff membrane of cellulose when grows in an appropriate nutrient solution. Fontana et al. claimed that such sort of information is more helpful for grade 2 and 3 burning ulcers and even for graftedskin as well [41]. Banerjee et al. 2010 assessed the Kombucha extract’s effective treatment on cutaneous wound healing in vitro condition [42].

The article "Histopathological and clinical evaluation of Kombucha tea and Nitrofurazone on cutaneous full-thickness wounds healing in rats: an experimental study" was retracted in 2016. Reasons: misconduct by an author; plagiarized text; compromised peer review; false authorship.

In this research the shaved skin of male mouse was incubated in a DMEM culture medium by grade technique at phase between fluid and air for 3 days. Various doses 50, 25 and 75% were evaluated. The results showed that the Kombucha extracts has dose-dependent wound contraction effects. Bayat et al. (2009) in Iran investigated the oral Kombucha tea on cutaneous wounds mast cells in rat, and the obtained results indicated that the total mast cells count decreased in tested group on 7-15th days [43].

## Conclusion

Our study suggested that the promotion of wound healing, whereas the difference with other studies is in the healing effectiveness of Kombucha which was compared with the control, received no treatment, group. For this, its healing effects were more obvious and considered to be faster. However, in this study due to comparison with Nitrofurazone healing effects, ascertained that such sort of fungus healing effects was approximately similar to Nitrofurazone ointment. Therefore, Kombucha should be considered as potential primary therapy in the emergency department. However, further studies are indicated in this important area of wound healing research to evaluate the clinical efficacy of these agents and to search for the mechanisms that explain their effects.

## Competing interests

The authors declare that they have no competing interests.

## Authors’ contributions

RS, FB and FAH participated in the histopathological evaluation, performed the literature review, acquired photomicrographs and drafted the manuscript and gave the final histopathological diagnosis. JJ performed sequencing alignment and manuscript writing. EH, MR, MR and RS edited the manuscript and made required changes. All authors have read and approved the final manuscript.

## Supplementary Material

Additional file 1 Comparison of wound contraction. Click here for file
